The article "The Clinical Application and Prospect of Smart Prenatal Care and Postpartum Recovery" was retracted in 2023. Reasons: unreliable results or conclusions; concerns about the data; concerns about the peer review; concerns about the citations.

# The Clinical Application and Prospect of Smart Prenatal Care and Postpartum Recovery

**DOI:** 10.1155/2021/3279714

**Published:** 2021-10-06

**Authors:** Chang Shu, Shumei Han, Linli Li, Peng Xu, Yule Bai

**Affiliations:** ^1^Department of Obstetrics and Gynecology, The First Hospital of Jilin University, Jilin University, Changchun, Jilin Province 130021, China; ^2^Department of Medical Administration, The First Hospital of Jilin University, Jilin University, Changchun, Jilin Province 130021, China

## Abstract

Scientific and technological advancement has increased the requirement for modern medical systems, leading to smartphone-based intelligent prenatal care and postpartum recovery. This kind of prenatal care and postpartum recovery including a remote monitoring system for fetal heart monitoring, blood glucose, and weight overcomes the restrictions of time and space and provides all-round, convenient, rapid, and accurate services to the medical systems, doctors, and pregnant women. This paper reviews the current research on intelligent medical services for pregnant women, particularly for prenatal care and postpartum recovery.

## 1. Introduction

Intelligent medical services refer to the integration of advanced science and technology and modern medical services to optimize the medical systems and realize remote monitoring, diagnosis, and treatment [1]. Intelligent medical service is crucial for check-ups during pregnancy. It provides a convenient and individualized service of home monitoring during pregnancy, recording and monitoring the situation of pregnant women and fetuses at any time. Aided by advanced auxiliary software, doctors can also view recorded indicators through a smartphone app to guide female health care throughout pregnancy and detect abnormal conditions in time, to achieve early detection, diagnosis, and treatment. In addition, regional medical information exchange and sharing can achieve remote consultation of difficult cases and for critically ill pregnant women. This can alleviate the problem of uneven allocation of medical resources. Furthermore, video conferences and online lectures enable doctors to expand their knowledge and improve their medical vision and skills at home. Therefore, in this digital era, intelligent medical service has gradually improved prenatal care and postpartum recovery, increasing the efficiency of medical services. The review shows that the application of intelligent medical services will bring epoch-making changes in the medical systems.

## 2. Prenatal Care during Pregnancy

Standardized prenatal examination can prevent and cure pregnancy complications as soon as possible, detect fetal abnormalities in time, evaluate the safety of pregnant women and fetuses, determine the time and mode of delivery, and ensure the safety of mothers and children to a greater extent [2, 3]. At present, prenatal examination in China is recommended in 6–13^+6^, 14–19^+6^, 20–24, 25–28, 29–32, 33–36, and 37–41 weeks (once a week). The disadvantage of this examination is that hospitals can only record indicators of pregnant women in the process of labor inspection, but cannot determine whether pregnant woman are under abnormal conditions. As a result, pregnant women are in the absence of professional monitoring except the birth examination; thus, doctors are unable to make timely assessment and treatment of abnormal conditions of pregnant women, and effective diagnosis and treatment of diseases can be delayed [4].

The situation is worse for some pregnant women with high-risk factors such as old age, obesity, and family genetic diseases. The probability of complications during their pregnancy is relatively high [5], and the frequency of labor examination should be greatly increased to prevent patients from missing the best time for diagnosis and treatment. However, frequent intensive care increases the time and effort of pregnant women due to line-ups at hospitals and travels to hospital. This will cause at least three serious problems. First, the high economic burden caused by the long-time monitoring of the patients will result in greater economic pressure on the patients. Since they often go to the hospital to see a doctor, they will also suffer from various psychological and physiological pressures. Second, hospitals cannot monitor every pregnant woman frequently because of the shortage of monitoring and inspection equipment and the limitation of some medical resources. The medical resources of primary hospitals are insufficient. In spite of abundant medical resources, high-level hospitals encounter such problems as too many patients can cause waste of both time and medical resources since most of them are unfamiliar with medical treatment procedures. Waste of time also leads to an amount of unnecessary trouble to patients and doctors. Third, many female patients face the double pressure from family and society. They tend to avoid medical treatment and conceal medical history, so doctors are unable to make a correct and timely diagnosis and treatment, delaying the best treatment opportunity. Most pregnant and lying-in women lack experience and professional knowledge. Even if they have precursor symptoms, they choose to rest and recuperate at home, thus missing the best opportunity for clinical intervention.

Therefore, it is significant to effectively carry out early disease detection, diagnosis, and treatment through incorporating intelligent technology into modern medical treatment [6]. This can facilitate early identification and early intervention of female pregnancy diseases, avoid the occurrence of complications, and relieve the economic and psychological pressure of patients and the urgent requirement for medical resources. Clinical applications of intelligent medical treatment are necessary to meet the requirement for remote monitoring of pregnant women in different environments.

## 3. Clinical Application of Smart Medical Service in Female Pregnancy

The introduction of the second child policy in China increases the number of high-risk pregnant women as well as the probability of adverse pregnancy outcomes. For these women, therefore, intelligent medical service undoubtedly becomes an indispensable medical choice. Many intelligent medical APPS (Mei pomelo, Chunyu doctor, baby tree gestation, and some WeChat small programs) emerged at the historical moment, and intelligent technology has also received greater attention and clinical application of [7] in the field of modern medical services. Pregnant women can obtain convenient medical services by perfecting their personal files, sharing information with hospitals, improving their knowledge of health care during pregnancy, and remotely monitoring fetal heart, blood glucose, weight, and so on [8–11].

### 3.1. Remote Monitoring System for Fetal Heart Monitoring

Fetal heart monitoring, one of the important means to monitor fetal status during pregnancy, continuously observes and records the dynamic changes of the fetal heart rate (FHR), evaluates the intrauterine safety situation of the fetus, and understands the relationship between the fetal heart, fetal movement, and contractions. In the past, pregnant women with fetal heart care needed to go to the hospital for regular examination. Due to the large number of patients and the long time spent, the patients usually had negative medical treatment experience. The outpatient fetal heart monitoring data were not conducive to preservation and analysis. However, thanks to the continuous development and application of Internet information technology in the medical field, Internet medical care has been adopted, creating new models of self-managed health care. For example, in recent years, the universal fetal remote monitoring system can carry out examination of the fetal heart and fetal movements at any time, monitoring the health status of the fetus and uploading the data to hospitals. This system runs through the Internet equipment composed of a central monitoring station, fetal monitor, and family fetal monitor and can identify the abnormal condition of the fetus in time and address it.

The specific operation procedures of the remote fetal heart monitoring system are as follows:

1. Establish the remote fetal heart monitoring system, composed of the mobile Doppler fetal heart monitoring instrument, the app of remote maternal and infant health care, and the electronic terminal of hospitals.
2. Establish a health file to collect and input the basic information of pregnant women in the maternal and infant app, including name, age, last menstruation, pregnancy and birth history, and previous medical history. This enables remote sharing, remote consultation for high-risk pregnant women, and online consultations.
3. Inform pregnant women for both the use of fetal heart examination and the significance of monitoring; guide pregnant women to count fetal movements in the early, middle, and late days; and upload the app for automatic interpretation and analysis. If abnormal monitoring occurs, the equipment will automatically alarm the electronic terminal of the hospital, and the data will be interpreted by the medical staff for intervention if necessary.

Godfrey R, Mugyenyi, and other researchers analyzed and evaluated the monitoring results of the remote fetal heart monitoring system and the effect of hospital fetal heart monitoring. They showed that there is no significant difference in the detection rate of normal and abnormal graphics between the two monitoring methods [12]. However, Liu Wei et al. used the remote fetal heart monitoring system in prenatal monitoring of early onset, finding that severe preeclampsia can increase the incidence of complications and perinatal outcome [13]. We can compare the monitoring results of the remote fetal heart monitoring system with those of traditional hospital fetal heart monitoring in terms of the relevant data of abnormal fetal heart, fetal movements, amniotic fluid, and umbilical cord. This comparison will indicate that the application of remote fetal heart monitoring can effectively reduce the incidence of abnormal prognosis of newborns and better protect the life safety of pregnant women and newborns. Therefore, the application of a remote fetal heart monitoring system can better protect the maternal and fetus, detect pregnancy complications as soon as possible, and decrease the inconvenience caused by the uneven distribution of medical resources. This is significant for the model innovation of maternity examination for pregnant women. However, there are still some shortcomings in this mode, such as nonstandard patient operation, delayed doctor-patient communication, and differences in equipment accuracy compared with conventional fetal heart rate monitoring. At present, although there are no adverse outcomes caused by incorrect interpretation of fetal heart rate monitoring, this latent danger exists and needs to be gradually improved in the future.

### 3.2. Remote Monitoring System for Blood Glucose and Weight

Gestational diabetes mellitus (GDM) is typical sugar intolerance, with such adverse outcomes as massive fetus, birth trauma, and perinatal complications. The risk of these consequences increases as mothers increase their fasting blood glucose levels. Artificial intelligence is an effective tool to help monitor and treat GDM.

The specific operation procedures of applying artificial intelligence to deal with GDM are as follows:

1. Establish the remote blood glucose monitoring system composed of mobile blood glucose monitor, app of remote health care for the maternal and infant, and the electronic terminal of hospitals.
2. Establish a health file to collect and input the basic information of pregnant women in the maternal and infant app, including name, age, last menstruation, pregnancy and birth history, height, weight, and previous medical history. This enables remote sharing, remote consultation for high-risk pregnant women, and online consultations.
3. Inform pregnant women in both the use of the system and significance of the blood glucose meter; guide pregnant women diagnosed with gestational diabetes to measure blood sugar six times a day (after getting up, two hours after each of the three meals every day, and before and in the middle of sleep every night). Record daily weights and upload them to the app for automatic interpretation and analysis. Abnormal blood sugar results will trigger automatic alarms at the hospitals' electronic terminal and be interpreted by medical staff who will give guidance for diet, exercise, and other aspects of life. The interaction mode of blood glucose and other data is shown in Figure 1.

Mercedes Rigla and other researchers have shown the feasibility and widespread acceptance of a remote blood glucose monitoring system [14]. Although multiple studies [15, 16] found that comprehensive diet and exercise guidance did not reduce the incidence of gestational diabetes, the intervention could reduce the birth rate of macrosomia and the proportion of cesarean sections. This reduction can decrease the rate of obesity and the incidence of cardiovascular and metabolic diseases in children in the future. The traditional follow-up method for gestational diabetes patients is to follow-up once a week in hospitals, which has caused a large burden to medical institutions. These problems can be addressed by intelligent telemedicine, which provides viable alternatives that ensure clinical guidelines for treatment while saving medical resources.

### 3.3. Online Prenatal Education and Postpartum Depression Assessment System

Prenatal education classes inform pregnant women of the preparation required during pregnancy and childbirth and of related complications, thus effectively helping prospective couples to prepare for parenthood. Research has shown that prenatal classes help reduce postpartum pain in mothers with first delivery, reduce the risk of postpartum depression (postnatal depression (PND)) [17], and reduce parental stress and anxiety symptoms. Over the past decade, in response to the increasing burden of the healthcare systems, advanced computer-based technologies were considered as an effective means to support healthcare consumers. Currently, smartphone applications are useful tools for spreading health information, and relevant analytic studies also show that smartphone-based interventions may reduce depression and anxiety [18, 19].

The specific operation process is as follows:

1. Establish the remote prepregnancy curriculum system: the server uploads prenatal health education recorded by medical staff, including prenatal nutrition education, prenatal guidance, abnormal laboratory indicators interpretation, prenatal precautions and related complications, postpartum nursing, breastfeeding, and psychological guidance.
2. Establish health files: collect and input basic information of pregnant women in the maternal and infant app, including name, age, last menstruation, pregnancy and birth history, height, weight, and previous medical history. This enables remote sharing, remote consultation for high-risk pregnant women, and online Q and A.
3. Form and guide the patient to supply the postpartum depression score, which enables assessment of postpartum depression indicators and intervention treatment if necessary.
4. Designated interventions, nursing of postpartum perineostomy and caesarean wounds, breastfeeding or artificial feeding, postpartum recovery, neonatal care (bath and touch), neonatal vaccination, and postpartum reproductive health. If the patient has an abnormality, articles will be sent through the software to provide corresponding guidance.

Ko Ling Chan et al. found that pregnant women with prenatal education through software had lower levels of postpartum depression and postpartum anxiety than those without prenatal education. They also found that the smartphone-based intervention was less effective than traditional face-to-face teaching, which may be related to the imperfect function of the software, and that maternal-related anxiety was not effectively decreased [20]. However, the intervention effectively reduced the use of medical resources and the cost of maternity examination. According to [8], the daily mood of patients with postproduction depression improved within eight weeks after the APP guidance. Given that patients with depressive symptoms without intervention tend to improve over time [21], we cannot confirm those patients' improvement results from the use of applications so that a large number of clinical trials are necessary in future research.

### 3.4. App-Based Pelvic Floor Functional Recovery System

Stress urinary incontinence is a common concern in women, which has a wide range of adverse effects on the quality of life and has significantly affected patients and society [22]. A growing body of epidemiological evidence suggests that the gestational prevalence of stress urinary incontinence is 18.6–60% and increases with age [23]. Pregnancy and childbirth can damage the nerve, connective tissues, and muscle tissues of the pelvic floor and perineum, thus being the main risk for stress urinary incontinence. Although pelvic floor damage from pregnancy and childbirth has been widely recognized, there is limited attention to the prevention and treatment of stress urinary incontinence in pregnant women.

The specific operation process of the app-based pelvic floor function recovery system is as follows:

1. Establish pelvic floor function recovery system: the server uploads the pelvic floor recovery training video recorded by the medical staff.
2. Establish health records to collect and input basic information on pregnant women in the APP of remote health care for mothers and children, including name, age, last menstruation, pregnancy history, height, weight, and past medical history. The patients were evaluated by color ultrasound of the pelvic floor.
3. Arrange reasonable training methods and frequency for different pelvic floor damage. A follow-up treatment is often arranged six weeks, three months, and six months after delivery.

At present, one of the effective treatment schemes for urinary incontinence is Kegel exercise [24]. In the past, supervising patients to recover pelvic floor function costs a large amount of manpower and material resources, and the rate of missing visits was high. However, with the popularity of mobile phones, mobile applications may offer great potential for providing health services and enhancing adherence to pelvic floor muscle training. One study of 123 adult women in Sweden showed a significant improvement in symptom severity and quality of life in the APP group, compared with those in the delayed treatment group [25]. Compared with the historical control group, the mobile phone group showed a significantly lower prevalence rate, and compliance was better [26]. Xiaojuan Wang et al. used app audio to guide women to pelvic floor muscle training for improving pelvic floor muscle strength, bladder neck mobility, and sexual function [27]. Simple Kegel exercise did not work well [28] for postpartum pelvic floor muscle recovery combined with pelvic floor physiological electrostimulation. However, due to the reduced time and cost, this method still has a positive role in the majority of maternal postpartum recovery. The advantages and disadvantages of smart prenatal care are shown in Table 1.

### 3.5. Intelligent Medical Care Associated with Pregnant Women and Novel Coronavirus Pneumonia (COVID-19)

Recently, Huiliang Wu conducted a web-based survey on Chinese pregnant women through the national online platform (BAMI National Maternity School) to investigate their self-protection behavior and attitude towards prenatal care during the pandemic. A total of 983 Chinese pregnant women completed the questionnaire survey. It was found that more than 80% of pregnant women took self-protection measures, such as wearing masks, washing hands, and isolation at home so as to avoid infection with severe acute respiratory syndrome. The survey show that, about 20% of the respondents are afraid of any form of consultation in the hospital, while more than 40% of the respondents are afraid of prenatal examination in the hospital. In addition, more than half of people considered or decided to cancel their inhospital prenatal examination and postpone their appointment. These behaviors and attitudes indicate that pregnant women are anxious and worried about the potential infection in the hospital environment. Considering the above difficulties and fear of other unknown factors in hospital visits, online prenatal care may be a better choice for pregnant women during this pandemic [29]. Hannakaisa Niela-Vile ´ *n* et al. reported heart rate variations, physical activity (step count), and life pressure changes (sleep duration) for known pregnant women during the COVID-19 outbreak in Finland and used a smartwatch to track all parameters. The feasibility of this approach to [30] is confirmed. Since the epidemic of COVID-19, the obstetric clinic of the Erwin Medical Center of Columbia University has begun to transform the maternity examination into a telemedicine mode. Inperson tests are necessary just when laboratory tests and color Doppler ultrasound examinations are necessary. This mode is not a clear indication of any benefit. The quality of virtual tests is related to the patient's own medical information acceptance. However, maintaining monitoring and routine intervention during the virtual appointment period can reduce the risk of exposure. However, the popularization of telemedicine during the pandemic still faces many challenges, such as information security, quality control, language communication, and hardware equipment. And, there are no reports that can provide relevant data to prove the advantages of smart medicine. But in any case, this can reduce the exposure to COVID-19, and the advantage is of no doubt [31]. At present, this follow-up method still needs to improve more testing items.

### 3.6. Improvement of Medical Experience of Pregnant Women in Areas with Uneven Allocation of Medical Resources

For pregnant women in remote areas with medical resources and lack of experience, doctors can guide pregnant women during pregnancy by uploading their weight changes, blood pressure monitoring, and laboratory tests, especially for pregnant women with high-risk factors (such as advanced pregnancy and intrahepatic cholestasis of pregnancy). These factors can contribute to the proper prolongation of gestational weeks, greatly reducing the premature birth rate, disability rate, and mortality rate of the fetus and greatly increasing the survival rate of pregnant women. This is of great significance to improve the quality of health care during pregnancy and promotes medical development in remote areas [28, 30, 32]. With the popularity of intelligent medical technology, any abnormal situation in pregnant women can be dealt with in time through intelligent medical care. For example, a fetal heart monitoring system can be used at any time when pregnant women feel abnormal fetal movements. The system will automatically record the monitoring results and scores and store them. Doctors can also get results in time, according to the results of online guidance or notification to the hospital. It can not only avoid unnecessary hospital commuting but also realize timely diagnosis and treatment for abnormal and serious conditions such as fetal intrauterine ischemia and hypoxia [32–35].

## 4. Epoch-Making Significance of Intelligent Medical Treatment to Implement Clinicians' Diagnosis and Treatment Activities

Recent years have witnessed the emergence of various smartphone apps, and the software for obstetricians is also being gradually developed and used. The apps are gradually facilitating clinicians and imperceptibly changing treatment patterns.

### 4.1. Yunsuan App

In the past work, obstetricians took the turntable to calculate the pregnancy period or paper and pen to predict the maternity date through calculation, which is time-consuming and laborious. Additionally, errors occur in artificial calculation, which is not intelligent enough. Pregnant calculation app is a small program in WeChat (the Yunsuan app and the following apps' icons are shown in Figure 2). It includes a series of functions such as estimated date of confinement and gestational age calculation, fetal growth and weight, growth labeling interpretation, fetal umbilical blood flow evaluation, Doppler evaluation of central cerebral artery, and cervical transparent layer. This provides strong support for clinicians in clinical work to calculate accurate gestational weeks, especially during outpatient visits. Additionally, the system helps reduce the risk of fetal growth, the risk of outpatient misdiagnosis, and missed diagnosis.

The advantages of this software are as follows. (1) The estimated date of confinement can be calculated through the last menstruation, head and hip diameter, and embryo transplantation date, to maximum avoid the weekly pregnancy calculation errors. (2) The fetal weight evaluation can use INTERGROWTH-21st samples of Chinese people, NICHD, Chinese University of Hong Kong, and Chinese semicustomized curves. More accurate assessment can be conducted for different groups. For example, the southern China recommends curve established by the Chinese University of Hong Kong. Assessment of the other three features is designed in accordance with the latest guidelines and large sample data. In all, pregnancy computing software provides quite strong support and convenience for clinicians.

### 4.2. Yousheng Think Tank

This is a birth defect-related software for doctor work, including literature process, lecture, courseware, guide consensus, expert consultation, medication consultation, and other modules. This software provides a variety of birth defect-related research progress and consensus guided by various birth defect-related diseases. Clinicians can gain knowledge and make progress at any time through this app. The app also set up an expert consultation platform with famous prenatal diagnostic experts throughout the country. When encountering difficult cases, regiment women can collate the relevant information and consult relevant experts, building a higher platform for clinicianism. The platform also provides better protection for guiding patients for further treatment.

### 4.3. Good Day

The software is the work platform for doctors from the first Hospital of Jilin University. Patients can be managed through mobile phone clients. Examination and laboratory results can be found on electronic medical records at any time in the medical group of patients' orders. Patients can be directed and managed anytime and anywhere, and online counselling will be open in the future. Any questions and puzzles arising from patients in the hospital can be exchanged on this platform. Especially when doctors are not in working hours, they can also deal with the patient's condition at any time, overcoming time and space barriers.

Besides the abovementioned apps, excellent intelligent medical software has been developed, such as medical pulse, clinical guidelines, and uterine contraction recorder. All these apps bring great convenience to the doctor's work. With the development of AI technology, various kinds of medical software will keep emerging, and there will be more comprehensive and intelligent software applicable to obstetrics in the future. The application of the software can improve the quality of medical treatment and the efficiency of diagnosis and treatment and reduce the rate of misdiagnosis and missed diagnosis. In addition, the system will improve the pattern of diagnosis and treatment, promoting the innovation of diagnosis and treatment methods. All of these achievements are of epoch-making significance.

## 5. Limitations and Prospects of Smart Medical Treatment

### 5.1. Limitations of Smart Care

Although the trend of replacing the traditional medical models with intelligent medical treatment has been unstoppable, the transformation will take a long time. China's intelligent medical care has developed continuously. While bringing us convenience, the service platform will inevitably encounter some problems.

1. When patients use intelligent medical systems, they need to improve their personal information and upload the results of each examination, which may involve some privacy data. If the data are not safely used with unreasonable management, it may infringe on the rights of patients and cause unnecessary harm to them.
2. The application of intelligent medical care is relatively simple, but accuracy cannot be guaranteed at present. This quality of this medical care remains to be improved in the presence of difficult cases.
3. Intelligent health care has not been accessible to those relatively backward areas.
4. Different from artificial medical treatment, intelligent health care is unable to carry on comprehensive barrier-free communication with the patient, easy to cause misdiagnosis and missed diagnosis.
5. Relevant legal systems have not been built up and perfected.
6. During the operation of relevant medical activities, due to the lack of professional knowledge, patients are unable to identify all kinds of emergencies and special situations like medical staff, which is more likely to cause measurement errors, and then there is the possibility of medical negligence. Therefore, more attention should be paid to the training of patients' professional knowledge, and more publicity and education videos should be added to the software to minimize such mistakes.

### 5.2. Prospects of Smart Medical Care

The problems in modern medical treatment, such as the regional imbalance of medical care and a lack of professional talents, can be alleviated by the wide application of intelligent technology. With the increasing understanding and application of intelligent medical care, and through the use of a portable or family fetal heart monitoring instruments, we can detect abnormal situations anytime and anywhere, providing timely and relevant diagnosis and treatment guidance [34]. This will significantly facilitate “early detection, early prevention, early diagnosis, and early treatment,” reducing the incidences, disability, and mortality of diseases, as well as the burden for society and families [36, 37]. In addition, the patient data obtained by smart medical treatment are more detailed and timely than the data obtained from the hospital follow-up. Through these statistics, more medical activities can be carried out, such as gestational diabetes mellitus, which can not only get the blood sugar data of each patient but also bind the data to the diet and make a comprehensive analysis. Moreover, all data are stored in the terminal server, which is more convenient for statistics and using, so it also shows potential research value.

This paper has systematically reviewed the integration of artificial intelligence with modern medical treatment and highlighted the direction of future research. Since intelligent medical treatment will inevitably become a trend in the medical field [38], further studies and applications are necessary for adaption to changes, solution to pertinent problems, improvement of medical services, and sustainable development of intelligent medical treatment.

First of all, there are great difficulties in the development of intelligent obstetric care. At present, it is very difficult to realize the full development of intelligent obstetric care because specialized examinations including color Doppler ultrasound and laboratory tests still need to be carried out in the hospital. Therefore, intelligent medical treatment should be used as a supplement to the existence of traditional treatment. This needs to abandon the shortcomings of traditional medicine and replace it with the intelligent medical model. At the same time, it should be combined with necessary traditional medicine. Secondly, the intelligent medical model still needs to be popularized and popularized. At present, there is endless software, there is no unified supervision and standards, and their therapeutic purposes and effects are different. Therefore, it needs to be more standardized.

## Figures and Tables

**Figure 1:** Data exchange mode through software of GDM.

**Figure 2:** The icons of apps above and below.

**Table 1:** The advantages and disadvantages of smart prenatal care.

	Prenatal care	Smart	Traditional
Fetal heart monitoring	Economic pressure	Low	High
	Time cost	Low	High
	Psychological pressure	Weak	Strong
	Data saving	Easy	Hard
	Measurement error	High	Low
	Fetal abnormalities found	Early	Late
	Portability	Strong	Weak
	Monitoring result	Same	Same

Blood glucose monitoring	Monitoring frequency	High	Low
	Incidence of macrosomia	Low	High
	Cesarean section	Less	More

Postpartum depression	Treatment effect	Good	Better
	Popularization difficulty	Easy	Hard
	Equipment accuracy	Low	High
	Depression and anxiety	Low	Lower

Pelvic floor rehabilitation	Treatment effect	Good	Better
	Lost follow-up rate	Low	High
